The article "Design of an Incremental Music Teaching and Assisted Therapy System Based on Artificial Intelligence Attention Mechanism" was retracted in 2023. Reasons: signs of a paper mill; suspected computer-generated content; unreliable results or conclusions; lack of ethics approval or compliance.

# Design of an Incremental Music Teaching and Assisted Therapy System Based on Artificial Intelligence Attention Mechanism

**DOI:** 10.1155/2022/7117986

**Published:** 2022-06-16

**Authors:** Dapeng Li, Xiaoguang Liu

**Affiliations:** ^1^Department of Music and Dance, Changzhi University, Changzhi, Shanxi 046011, China; ^2^Changzhi Medical College, Changzhi, Shanxi 046011, China

## Abstract

With the continuous updating and advancement of artificial intelligence technology, it gradually begins to shine in various industries, especially playing an increasingly important role in incremental music teaching and assisted therapy systems. This study designs artificial intelligence models from the perspectives of attention mechanism, contextual information guidance, and distant dependencies combined with incremental music teaching for the segmentation of MS (multiple sclerosis) lesions and achieves the automatic and accurate segmentation of MS lesions through the multidimensional analysis of multimodal magnetic resonance imaging data, which provides a basis for physicians to quantitatively analyze MS lesions, thus assisting them in the diagnosis and treatment of MS. To address the highly variable characteristics of MS lesion location, size, number, and shape, this paper firstly designs a 3D context-guided module based on Kronecker convolution to integrate lesion information from different fields of view, starting from lesion contextual information capture. Then, a 3D spatial attention module is introduced to enhance the representation of lesion features in MRI images. The experiments in this paper confirm that the context-guided module, cross-dimensional cross-attention module, and multidimensional feature similarity module designed for the characteristics of MS lesions are effective, and the proposed attentional context U-Net and multidimensional cross-attention U-Net have greater advantages in the objective evaluation index of lesion segmentation, while being combined with the incremental music teaching approach to assist treatment, which provides a new idea for the intelligent assisted treatment approach. In this paper, from algorithm design to experimental validation, both in terms of accuracy, the operational difficulty of the experiment, consumption of arithmetic power, and time cost, the unique superiority of the artificial intelligence attention-based combined with incremental music teaching adjunctive therapy system proposed in this paper can be seen in the MS lesion segmentation task.

## 1. Introduction

The development of artificial intelligence and brain science complement each other; for example, the neural network in artificial intelligence theory mainly draws on the connection principle of neurons in the biological brain, and the design of a deep convolutional neural network mainly refers to the convolutional structure and multilayer structure in brain vision, and the attention mechanism of the biological brain also inspires people to think about the attention module in a neural network [1]. The development of brain science has promoted the innovation of artificial intelligence technology, but how to apply the artificial intelligence technology represented by the deep neural network to the field of brain science to realize the automatic prevention and diagnosis of neurological diseases is an important scientific research topic. Meanwhile, in the process of incremental music teaching, it can be found that music also prompts neuronal activity in the biological brain in a form that can be referred to as the attentional adjustment mechanism in brain vision.

The article "Design of an Incremental Music Teaching and Assisted Therapy System Based on Artificial Intelligence Attention Mechanism" was retracted in 2023. Reasons: signs of a paper mill; suspected computer-generated content; unreliable results or conclusions; lack of ethics approval or compliance.

With the rapid development of artificial intelligence technology represented by deep neural networks, it is possible to achieve automatic and accurate segmentation of MS lesions based on MRI [2]. The realization of automatic and fast accurate MS lesion segmentation can not only reduce the burden of manual segmentation of MS lesions by experts, save the time and energy of experts in analyzing patients' conditions, and reduce the incorrect diagnosis due to subjective factors of experts, but also, because MS lesions show diffuse and multiplicity in imaging, it is difficult for inexperienced doctors to identify them accurately, and the realization of automatic and accurate MS lesion identification can to a certain extent, the automatic and accurate identification of MS lesions can assist in the diagnosis of MS by inexperienced physicians, which is conducive to the promotion and use in medically underdeveloped areas [3]. Therefore, studying the automatic segmentation model of MS lesions and improving the segmentation accuracy and generalization performance of the MS lesion segmentation model can help physicians quickly and accurately diagnose patients' conditions and promote effective treatment and etiological discovery of MS. To track the disease progression in the brain, multimodal neuroimaging techniques are mainly used in clinical practice. For example, positron emission computed tomography imaging images can reflect the metabolic information of the organism at the molecular level; computed tomography imaging reflects the tissue information of the human brain through the spatial distribution of X-ray absorption; magnetic resonance imaging can reflect the information of soft tissues such as human organ disorders and tissue lesions, which can well display the anatomical structure and lesion information; among them, MRI is based on different repetition times; MRI is divided into T1 image, T2 image, and FLAIR image according to different parameters such as repetition time, echo time, and inversion time.

The article "Design of an Incremental Music Teaching and Assisted Therapy System Based on Artificial Intelligence Attention Mechanism" was retracted in 2023. Reasons: signs of a paper mill; suspected computer-generated content; unreliable results or conclusions; lack of ethics approval or compliance.

The basic design principle of layer-by-layer abstraction of convolutional neural networks dictates that deeper feature layers of convolutional neural networks will have larger perceptual fields and higher semantic levels and focus more on overall semantic information and larger objects. However, segmentation networks using ordinary convolution usually do not focus on shallow features with detailed semantic information, so many studies have introduced null convolution and multiscale context fusion modules to integrate semantic information at different scales, focusing on both larger objects and overall information, as well as smaller objects and detailed information, and can combine contextual information to make more accurate inferences [4]. For the lesion segmentation task, the context module can capture not only the lesion information but also the pathological information related to the lesion from the tissues surrounding the lesion.

When we look at a picture, our eyes will only focus on a certain pattern in the picture instead of the whole picture, and the human brain will only focus on a certain part at this time; i.e., the human brain does not pay attention to each part of the whole picture in the same way, which is the core idea of the attention mechanism. Introducing the attention module in the network model of MS segmentation can enhance the representation of lesion features. In this paper, we propose a cross-dimensional attention mechanism, aiming at capturing the lesion information of multiple sclerosis in MRI data from multiple dimensions and improving the generalization ability of the model.

For multiple sclerosis lesions, the presence of a lesion at a certain location may lead to changes in the surrounding tissues, so the voxels around the lesion have certain pathological information. To make full use of the surrounding contextual information, a 3D context-guided module is designed, which uses convolutional operations to obtain the higher-order local information, while the surrounding information is obtained based on inflated convolutional operations [5, 6]. The final output will combine the input low-level local information, the obtained high-level local information, and the surrounding information. Also, considering the disadvantages of the null convolution with the tessellation effect and the possibility that the long-range information is irrelevant to the task, Kronecker convolution is introduced in the design of the above module to better capture the surrounding contextual information.

The article "Design of an Incremental Music Teaching and Assisted Therapy System Based on Artificial Intelligence Attention Mechanism" was retracted in 2023. Reasons: signs of a paper mill; suspected computer-generated content; unreliable results or conclusions; lack of ethics approval or compliance.

In the process of combining incremental music instruction with complementary therapy, MS patients have different individual abilities to perceive, discriminate, compose, and express music based on music, as demonstrated by their mastery of a variety of basic musical elements, such as intensity, tempo, beat, timbre, and common structures, as well as their ability to express their thoughts and feelings directly through artistic forms such as singing, playing, improvisation, and creative practice. The individual can use singing, playing, improvisation, creative practice, and other art forms to directly express their thoughts and feelings, and to process, create and understand the high meaning of sound. Multiple Intelligences (MI) theory is used to address the differences between individual patients, both in terms of neurological differences between patients and in terms of helping them to develop effectively and holistically so that those who are impaired in one area of intelligence can fully recover [7]. When designing a music teaching-assisted therapy context, the physician will take into account various factors of the patient, from the perspective of mobilizing the patient's interest in music learning to the main penetration of the work teaching context creation, with the help of visual and imaginative methods or means of creating the context, reproducing the mood of the work, visualizing the abstract music, making the hard knowledge interesting, realizing the full activity of the neurons in the brain, obtaining more fully the lesion Peripheral pathological information to promote autoimmunity and subsequent therapeutic work.

The most important differences between the artificial intelligence attention mechanism and the incremental music teaching method and the traditional treatment method are the feature extraction stage. Depth features not only reduce the errors caused by the manual feature extraction process but also have better learning ability and differentiation ability.

Multiple lesions are diseases of the brain, and when designing automatic segmentation models, they often operate on the whole brain, while different patients, with multiple sclerosis, have different lesion locations, sizes, numbers, and shapes [8]. Spatial details are often lost in higher-order output mappings due to cascaded convolution and activation function nonlinearity. Meanwhile, the attention mechanism is proposed for the deep learning black box mechanism, which can effectively solve the problems of poor interpretability and weak generalization ability of convolutional neural networks.

The article "Design of an Incremental Music Teaching and Assisted Therapy System Based on Artificial Intelligence Attention Mechanism" was retracted in 2023. Reasons: signs of a paper mill; suspected computer-generated content; unreliable results or conclusions; lack of ethics approval or compliance.

## 2. Method

### 2.1. Design

To better evaluate the validity of the model proposed in this study, five evaluation metrics were used: dice overlap, positive predictive value, true false positives of lesions, false positives of lesions errors, and absolute volume difference. Finally, the overall evaluation score was used for the final evaluation.

### 2.2. Dataset

This study used the SBI2015FMI longitudinal multiple sclerosis dataset to experiment. The dataset was divided into a total of three groups, the training set, test set A, and test set B. The training set consisted of five patients, four of whom had four-time acquisition points and the fifth patient had five-time acquisition points. Test set A consisted of 10 patients, 8 of which had 4-time acquisition points, 1 had 5 acquisition points, and 1 had 6-time acquisition points. Test set B had 4 patients, 3 of whom had 4-time acquisition points and 2 had 5-time acquisition points.

### 2.3. Experimental Method

The ACU-Net proposed in this study was implemented in Python language using the Keras library based on the tensor flow backend. All experiments were conducted on a workstation with a GTX 3090 with 12 GB RAM and an Ubuntu system. The SGD algorithm was used as an optimizer to train the network, where the learning rate, decay coefficient, and momentum were taken as 0.05, 10^−4^, and 0.9, respectively. The image size of all MRIs had a fixed size of 180∗220∗180 voxels, which were cropped to 160∗192∗160 during the training process. A four-channel convolutional neural network was constructed using the four provided modalities: FLAIR, Tl, T2, and PD, and was experimentally trained for 80 cycles. The module cleverly integrates Kronecker convolution-based contextual information capture, aggregation of the channel and spatial information, 3D voxel features, and 2D pixel features. The integration of this module into the decoding phase of the U-shaped network enables the model to capture lesion information from multiple dimensions, multiple channels, and multiple fields of view. For the images used in the experiments, four types of feature extraction were used, which were extracted morphological features, grayscale difference statistics, grayscale gradient coeval matrix, and wavelet transform features, and then the above features were serially fused, and the Lasso algorithm was used for feature selection [9].

The grayscale difference statistical feature uses the grayscale difference between the grayscale of each pixel point of the image sample and the neighboring pixel points to describe the texture features, and it achieves the elimination of interfering pixels by approximating the pixel values of similar points in the image. Let (*x*, *y*) be a point in the image; then the grayscale difference value between this point and the other similar points (∆*x* + *x*, ∆*y* + *y*) is *g*∆(*x*, *y*) = *g*(*x*, *y*) − *g*(*x*+∆*x*, *y*+∆*y*), where *g*∆ is the grayscale difference [9]. If the image gray level is *m*, let the point (*x*, *y*) move on the given image to obtain the histogram of *g*∆(*x*, *y*), and from the histogram, the probability that *g*∆(*x*, *y*) takes the value of *p*(*k*) when the histogram is relatively flat means that the picture texture is more detailed. On this basis, some feature values can be used to quantitatively represent the features of the image, and the commonly used feature descriptors are contrast, angular direction second-order moment, mean value, entropy, etc.

The article "Design of an Incremental Music Teaching and Assisted Therapy System Based on Artificial Intelligence Attention Mechanism" was retracted in 2023. Reasons: signs of a paper mill; suspected computer-generated content; unreliable results or conclusions; lack of ethics approval or compliance.

The grayscale gradient cooccurrence matrix is a method that uses the pixel grayscale and grayscale variation of an image to jointly describe the texture features of an image, which combines the gradient information of an image with the grayscale cooccurrence matrix, i.e., the statistical distribution of the grayscale of pixels and the edge gradients are united, and it better reflects the details and variations of the texture features of an image.

The data set was imported using R software, and the data set was randomly divided into a training set and a test set in the ratio of 7 : 3 using a random sampling method with put-back [10]. In the training set, the above clinical and morphological characteristics were included in a multi-factor logistic regression analysis, the age of patients (*β* = −0.029, OR = 0.97, *P* = 0.04), MS height (*β* = 0.485, OR = 1.62, *P* < 0.001), MS tumor neck width (*β* = −1.055, OR = 0.35, *P* < 0.001), A1 dominance sign (*β* = 0.675, OR = 1.96, *P* = 0.02), and MS irregularity (*β* = 1.464, OR = 4.32, *P* < 0.001) were independent risk factors for MS in front traffic. Specific information is shown in Table 1.

In a multifactorial regression model, the contribution of each independent risk factor to the dependent variable can be derived, the level of each influential factor is assigned a score, and finally, the conversion relationship with the probability of MS occurrence is derived, which leads to the predictive value of MS. Columnar graphs transform complex regression equations into visual graphs, making the prediction model more intuitive, easy to read, and practical for patient assessment, so they are becoming more and more widely used in clinical practice and research. Clinical decision curves (DCA curves) are another method that has emerged in recent years to evaluate the effectiveness of logistic prediction models. Plotting the ROC curve and comparing the area under the curve AUC often focus primarily on the accuracy, sensitivity, and specificity of the model; however, in a clinical work, the clinical decisions performed on patients with the aid of this predictive model can be affected by false negatives and false positives of the model [11]. Many studies have introduced null convolution and multiscale context fusion modules to integrate semantic information at different scales, focusing on both larger objects and overall information as well as smaller objects and details, and being able to combine contextual information to make more accurate inferences. For the lesion segmentation task, the context module can capture not only the lesion information but also the pathological information related to the lesion from the tissues surrounding the lesion. Relying solely on the ROC curve to evaluate the predictive model, the clinical benefit that patients receive because of the model is often not better reflected. Clinical decision curves can reflect the net clinical benefit (i.e., the net benefit rate after subtracting the benefit from the harm) for patients at a specific set of thresholds. Using the results from the Logistic model described above, the DCA curve is plotted in Figure 1, which shows that the model curve created by logistic regression is significantly higher than the backward-sloping reference line, which is positive, and that the predictive model has a better net patient benefit.

The article "Design of an Incremental Music Teaching and Assisted Therapy System Based on Artificial Intelligence Attention Mechanism" was retracted in 2023. Reasons: signs of a paper mill; suspected computer-generated content; unreliable results or conclusions; lack of ethics approval or compliance.

Combining the above evaluation indexes, we can see that the column line graph prediction model established by applying the traditional logistic regression can perform the prediction of MS risk better.

### 2.4. Results

To improve the predictive power of a model, we can generate many classification trees and later combine the results of these classification trees to improve the model performance, which is called random forest. A random sampling of both data and predictive features improves not only the model performance but also the generalization ability of the model. Ranking the magnitude of the impact of features on the improvement of the Gini index, we can see that in the random forest model, MS height, MS neck width, and the patient's age have a greater impact on MS rupture. Using the overall error rate as a criterion, the final optimal size of the tree in the random forest model was 116. Validating this random forest in the test set, the following results were obtained: the area under the ROC curve (AUC) was 0.733 (95% CI: 0.642-0.824), with an optimal cutoff value of 0.616. At this cutoff value, the accuracy of prediction in the test set was 0.677 (the accuracy of prediction in the test set at this cutoff value was 0.677 (95% CI: 0.587-0.758), sensitivity was 0.736, specificity was 0.596, and the Kappa value of consistency test was 0.334). Although the AUC was improved compared with the classification tree model, there was no significant improvement in the accuracy and other indicators [12].

The article "Design of an Incremental Music Teaching and Assisted Therapy System Based on Artificial Intelligence Attention Mechanism" was retracted in 2023. Reasons: signs of a paper mill; suspected computer-generated content; unreliable results or conclusions; lack of ethics approval or compliance.

In this model building, the training set, as well as the test set, is divided as before. Afterward, a feedforward neural network with 2 hidden layers was derived in the training set. After applying the model to the test set, the area under the ROC curve was calculated with an AUC of 0.733 (95% CI: 0.653-0.813) and an optimal cutoff value of 0.500, at which the sensitivity of the model was 0.736 and the specificity was 0.731. Similarly, we also compared the ROC curve of the traditional logistic regression model with that of the artificial neural network prediction model [13]. There is also no statistical difference between the two models, and they have similar model performance.

The MSO-Net network designed in this paper consists of six modules: a convolutional module for feature extraction, four edge output modules for obtaining segmentation results at different levels, and a fusion module for integrating these segmentation results. The convolutional module is mainly used for image coding and feature extraction. To obtain better feature extraction performance with limited training samples, we choose the current mainstream convolutional neural network and modify the backbone after training to build the convolutional module. For the MSO-VGGNets series network, we make two minor adjustments to build the convolutional module. Taking MSO-VGG19BN as an example, we first remove the fully connected layer at the end of the VGG19BN network. The fully connected layer can only accept a fixed size input, and it will not work once the image size changes [14]. By removing the fully connected layer, the proposed network can accept images of any size as input. In addition, since the fully connected layer discards the spatial relationship between pixels, it is also meaningless for subsequent resolution recovery. Second, we remove the maximum pooling layer of the last convolutional block of VGG19BN to maximize the resolution of the last feature map [15]. For the MSO-ResNets family of networks, taking the MSO-ResNet50 network as an example, for the same purpose, we remove the global mean pooling layer, the fully connected layer, and the softmax activation layer of the last ResNet50. After the adjustment, the convolutional modules all retain five convolutional blocks, i.e., convolutional block 1–convolutional block 5.

### 2.5. Incremental Music Teaching

The combination of contextual teaching and artificial intelligence attention theory makes the assisted treatment system more relevant, and the design of the treatment content more fully takes into account the patient's reality. By analyzing the characteristics of patients' multiple intelligences from the perspective of multiple intelligence theory, doctors combine and consider the characteristics of different bits of intelligence to create teaching contexts that correspond to their intelligence characteristics, which is more relevant to the implementation of treatment content and the goal of cultivating patients' intelligence and truly reflects the recovery-oriented music therapy [16]. When designing music teaching-assisted therapy situations, doctors will fully consider various factors of the patient, from the perspective of mobilizing the patient's interest in music learning works the main penetration of teaching situation creation, with the help of intuitive and visual methods or means of creating situations, reproduce the mood that the work wants to express, visualize abstract music, make the hard knowledge interesting, realize the full activity of neurons in the brain, more fully obtain the pathological information around the lesion, and promote autoimmunity as well as the subsequent treatment work. In the previous paper, the eight teaching strategies proposed by the music contextual teaching model developed by multiple intelligence theory were theoretically analyzed, but this is only the theoretical support, to further study the implementation of “patient development-based” “creating teaching contexts to cultivate patient intelligence”; in addition to further study the implementation of “patient development-oriented” “creating teaching contexts to cultivate patients' intelligence,” an experimental study on the contextual teaching-assisted treatment in junior high school based on multiple intelligence theory was conducted.

The article "Design of an Incremental Music Teaching and Assisted Therapy System Based on Artificial Intelligence Attention Mechanism" was retracted in 2023. Reasons: signs of a paper mill; suspected computer-generated content; unreliable results or conclusions; lack of ethics approval or compliance.

The strategy of creating authentic natural situations is based on the characteristics of natural observation intelligence. Natural observational intelligence is the ability of an individual to identify various organisms and be sensitive to the characteristics of nature and classify and use the environment. It is used to identify the characteristics of plants, animals, and things in the environment. Naturalistic observation intelligence is closely related to life and lifestyle in the natural world [17]. By creating the true context, the patient's natural observational intelligence can be developed and used to assist in treatment.

### 2.6. Analysis

MS lesions are widely distributed with large variations in shape and size, and capturing pathological information from three-dimensional space alone is insufficient. In this chapter, based on the previous chapter, we focus on the attention mechanism applicable to MS lesion segmentation and propose a multidimensional cross-attention U-Net. In this model, a cross-dimensional cross-attention mechanism is introduced for capturing pathological information in multiple dimensions and multiple channels [18]. Also, a multidimensional feature similarity module is introduced to improve the remote dependence of the model in multidimensional space. Experiments are conducted on the ISBI2015MS lesion dataset, and the experimental results show that the proposed model achieves better segmentation accuracy than existing methods.

## 3. Results

### 3.1. Patient Enrollment

The inclusion criteria were as follows: (1) the patient had a pathological diagnosis of EOC between January 2010 and February 2019; (2) the patient had an MRI scan four weeks before the gynecologic procedure; (3) the patient had the following four cross-sectional MRI sequences: fast spin-echo T2-weighted fat suppression imaging (T2WIFS), diffusion-weighted imaging (DWL with diffusion gradient factor b of 0 and 600 s/mm^2^, 0 and 800 s/mm^2^, or 0 and 1000 s/mm^2^), apparent diffusion coefficient (ADC), and delay-period enhanced T1-weighted fat suppression imaging (CE-T1WI). The exclusion criteria were as follows: (1) patients had undergone gynecological surgery and/or chemotherapy before MRI scanning, (2) patients did not have a clear histopathological diagnosis, and (3) patients have poor MRI quality (images with artifacts failing to outline tumor ROI regions). After exclusion and screening, a total of 305 patients were enrolled in this multicenter study, and the specific clinical information of the enrolled patients can be found in Table 2 [19]. Of these 294 patients, 144 patients from clinical centers A-B were classified as the training set, the remaining 75 patients were classified as the internal test set, and 75 patients from clinical centers C-H 75 patients were classified as the external test set.

### 3.2. Model Validation

For each NMR sequence, we construct a separate model. The Pearson correlation coefficients of all the features extracted from the sequence are calculated, and a Pearson correlation matrix is constructed based on this. The Pearson correlation coefficients of feature x and feature rare are calculated as*s*(*θ*; *t*) = *βe*^−*a*(*t* − *θ*)^2^^cos[2*πf*_*c*_(*t* − *θ*) + *ϕ*], where *θ* = [*β*, *a*, *τ*, *f*_*c*_, *ϕ*] is the number of samples, *τ* is the feature mean, *f*_*c*_ is the center frequency of the signal, *ϕ* is the phase of the wave, *β* is the amplitude coefficient [20], and *a* is the bandwidth factor; the absolute value of the Pearson correlation coefficient is between 0 and 1, and the larger the value, the stronger the correlation between the two features. The higher the value, the stronger the correlation between the two features, and the positive or negative sign of the correlation coefficient represents a positive or negative correlation, as shown in Figure 2. For the pairs of features with Pearson correlation coefficients greater than 0.9, we calculate their average Pearson correlation coefficients with other features and remove the larger one as a redundant feature.

The article "Design of an Incremental Music Teaching and Assisted Therapy System Based on Artificial Intelligence Attention Mechanism" was retracted in 2023. Reasons: signs of a paper mill; suspected computer-generated content; unreliable results or conclusions; lack of ethics approval or compliance.

We validated the diagnostic performance of the model on the internal (*N* = 75) and external (*N* = 75) test sets, respectively, and evaluated the performance of the model using the subject characteristic curves and the corresponding area under the curves.

### 3.3. Model Performance

As described previously, for each MRI sequence (T2WIFS, DWI, ADC, and CE-T1WI) of each patient, we extracted a total of 851 features from the manually outlined VOI. We removed the redundant features with a threshold of 0.9 and kept the top 4 features after mRMR sorting for model construction. The features used in different models and the corresponding weights can be seen in Table 3. It can be seen that the sphericity, which is a shape feature, is retained in all three models, DWI, ADC, and CE-T1WI, and is the only remaining feature in the ADC model. In addition, it is worth noting that all features are wavelet features except for the sphericity and a gray-scale travel matrix feature from the original image in the T2WIFS model [21].

The relative performance of the four unimodal models on the training, internal, and external test sets showed that the AUCs of the T2WIFS, DWI, ADC, and CE-T1WI models on the training set were 0.84, 0.93, 0.96, 0.95, and 0.87, respectively. In the external test set, the DWI model has the highest AUC of 0.94, while the other three models are 0.91, 0.86, and 0.88, respectively [22].

In addition, we constructed a mild-hybrid model based on the three MRI modes of T2WIFS, DWI, and ADC using the linear model, and the AUC values of the mild-hybrid model compared with the hybrid model are shown in Figure 3. The AUC values of the mild-hybrid model on the internal and external test sets were 0.782 and 0.834, respectively, with comparable accuracy to that of the hybrid model. Cross-attention across multiple dimensions can capture not only three-dimensional spatial pathological information but also three-dimensional through-truth information and two-dimensional spatial and channel-domain pathological information, which is beneficial to improving the model's ability to identify microscopic lesions. The results show that there is no significant difference between the ROC curves of the two (corpse = 0.06 on the internal test set and corpse = 0.15 on the external test set) [23].

The article "Design of an Incremental Music Teaching and Assisted Therapy System Based on Artificial Intelligence Attention Mechanism" was retracted in 2023. Reasons: signs of a paper mill; suspected computer-generated content; unreliable results or conclusions; lack of ethics approval or compliance.

The performance of the hybrid models built based on automatic outlining VOI was compared on the training set, internal test set, and external test set, and all three hybrid models (linear model, support vector machine, and decision tree) did not perform as well as the internal test set on the external test set. Among them, the hybrid model based on the linear model has the best overall performance, with AUC values of 0.813, 0.772, and 0.763 on the training set, the internal test set, and the external test set, respectively [24].

### 3.4. Weight Sharing

Weight sharing is a widely adopted strategy in deep learning, which can reduce model parameters and effectively avoid overfitting problems. We compare the performance of the model when multiple NMR modal feature extractors share and do not share weights. The performance of the model without weight sharing is better than that with weight sharing (AUC 0.8780.828). Weight sharing implies that the same feature extractor is used for different MRI modalities; however, the performance of ovarian tumors on T2WIFS, ADC, and CE-T1WI images is so different that using weight sharing for the same feature extraction is a less reasonable choice [25]. In contrast, if weight sharing is not used, each feature extractor can be adaptively adjusted to extract more features unique to their respective modalities. Moreover, SquzzeNet is a lightweight network with a small number of parameters, and using SquzzeNet pretrained with the ImageNet dataset for feature extraction also largely avoids overfitting, thus greatly reducing the need for weight sharing in the model.

To investigate the effect of different range sizes of contextual information on the model, we use different values of *c* to train the model. *c* = 0 indicates that the range of contextual information used is 0; i.e., the model has no C-MPL added. Models with C-MPL added (*c* > 0) all perform better than those without (*c* = 0), which indicates the effectiveness of C-MPL. As the value of *c* increases from 0, the model performance increases and peaks at *c* = 5, after which the model performance starts to decrease [26]. Too small a *c* value limits the utilization of background information, while too large a *c* value causes the model to consider too much irrelevant background information in prediction, making the target example less weighted and the model prediction performance decreases.

The article "Design of an Incremental Music Teaching and Assisted Therapy System Based on Artificial Intelligence Attention Mechanism" was retracted in 2023. Reasons: signs of a paper mill; suspected computer-generated content; unreliable results or conclusions; lack of ethics approval or compliance.

We analyzed the effect of different *R* values (*R* = 1, 2, or 3) on the MA module. The model achieves the best-integrated prediction performance when *R* = 3, at which time the AUC is 0.878, the accuracy is 0.827, and the F1 value is 0.875. The *R* value represents the number of neurons in the middle layer of the MA module, and since the inputs to the MA module are unimodal features of three NMR modes, an *R* value of 3 indicates that no dimensionality reduction is performed in the middle layer, and conversely, when *R* is less than 3, it indicates that the middle layer undergoes dimensionality reduction operation [27]. In the original SENet, the purpose of performing the dimensionality reduction operation is to reduce the model complexity. However, considering the very limited number of modalities used in our proposed model, this dimensionality reduction operation may narrow the pathways of the network and restrict the flow of information, thus leading to a degradation of the network model performance.

## 4. Discussion

The results of the segmentation of each network model on the ISBI2015MS lesion segmentation test set. From this table, it can be seen that 3DU-Net has the worst segmentation performance. Guided by the idea of coding and decoding of 3DU-Net, the ACU-Net model designed based on the context-guided module and the three-dimensional spatial attention model achieved certain segmentation results, based on which, further optimization was proposed to obtain the cross-attention mechanism across dimensions of MA CU-Neil network; as can be seen from the table, the PPV value and LFTP value of the model are optimized and the comprehensive evaluation value SC value is improved. With the addition of the multidimensional similarity feature module, the LFPR index of the network model MACU-Net2 is further improved, and at the same time, the LTPR value is further optimized, and the comprehensive evaluation value reaches 92.61 [28]. This indicates that the proposed module is effective and can well improve the accuracy of the convolutional neural network model for segmenting MS lesions.

To segment the model to better capture the pathological information of multiple sclerosis, a cross-dimensional cross-attention mechanism is proposed in this paper, which is an improvement on the contextual attention U-Net proposed in Chapter 3 and mainly optimizes the attention module of the model. The same as the contextual attention U-Net, this section introduces the cross-dimensional cross-attention based on cross-dimensional cross-attention used to connect the low-order features and high-order features of the U-Net [29]. The strategy of creating authentic natural situations is based on the characteristics of natural observation intelligence. Natural observational intelligence is the ability of an individual to identify various organisms and be sensitive to the characteristics of nature and classify and use the environment. We use naturalistic observation intelligence to identify the characteristics of plants and animals and various things in the environment. The difference is that cross-attention across multiple dimensions can capture not only 3D spatial pathology information but also 3D through-truth information and 2D spatial domain and channel domain pathology information, which is beneficial to improve the model's ability to identify microlesions. The excellent performance on the ISBI2015 longitudinal MS lesion dataset indicates that the proposed multidimensional attention U-Net is effective and feasible.

The article "Design of an Incremental Music Teaching and Assisted Therapy System Based on Artificial Intelligence Attention Mechanism" was retracted in 2023. Reasons: signs of a paper mill; suspected computer-generated content; unreliable results or conclusions; lack of ethics approval or compliance.

As a whole, the accuracy of the DenseNet121 model under full training has a small decrease compared to training the last convolutional block and fully connected layers, which indicates that the number of feature map channels is increasing while the size of the feature map is decreasing in the network, and although multiple layers of features are reused, it is possible to introduce noise or lose features [30]. In addition, the fine-tuned model using the public dataset works better than not using the public dataset, demonstrating that by reducing the interdomain variation, the accuracy in practical classification can be improved. Although the Inception v3 model achieves better results in method III, overall, the results of migration learning are inferior compared to traditional machine learning in terms of accuracy, the operational difficulty of experiments, consumption of computing power, and time cost.

## 5. Advantages and Limitations

In this paper, we introduce a multidimensional cross-attention module based on the study of contextual attention U-Net networks for MS lesions of this spatial multiplicity and combine it with incremental music teaching to assist treatment, which cleverly integrates Kronecker convolution-based contextual information capture, aggregation of the channel and spatial information, three-dimensional voxel features, and two-dimensional pixel features aggregation. The integration of this module into the decoding phase of the U-shaped network enables the model to capture lesion information from multiple dimensions, multiple channels, and multiple fields of view. In addition, a multidimensional feature similarity module is introduced to apply the module to the underlying layer of the U-shaped structure through multidimensional positional correlations, enabling the model to capture multidimensional remote dependencies. The superiority of the proposed multidimensional attentional U-Net for the MS lesion segmentation task is validated on the ISBI 2015 challenge dataset by comparing it with other and publicly published MS lesion segmentation models.

The article "Design of an Incremental Music Teaching and Assisted Therapy System Based on Artificial Intelligence Attention Mechanism" was retracted in 2023. Reasons: signs of a paper mill; suspected computer-generated content; unreliable results or conclusions; lack of ethics approval or compliance.

In terms of the generalization ability of the model, on the one hand, only one MS lesion segmentation dataset was used, and its data volume is not yet large, and the distribution of its data is hardly representative of all MS lesion types, which leads to the bias of the model in practical applications. On the other hand, this experiment was conducted using a publicly available dataset, which still has a certain gap from the actual clinical dataset.

## 6. Future Research Directions

From the perspective of network model design, on the one hand, the proposed network model requires a large number of hyperparameters requiring a lot of manual time for optimization, and some adaptive segmentation models should be tried in the future to automatically optimize the hyperparameters. On the other hand, the MS segmentation model is designed based on three-dimensional space. The fine-tuned model using the public dataset works better than not using the public dataset, demonstrating that by reducing the interdomain variation, the accuracy in practical classification can be improved. The three-dimensional network model requires a large number of parameters, which inevitably requires a large amount of time for a large number of calculations during training, which requires a high hardware configuration as well as a large amount of power consumption. This requires a high hardware configuration and a lot of power consumption. In the future, we will optimize the training efficiency to ensure the accuracy of the network while the lightweight network model reduces the complexity of the model and lowers the training cost [31]. In conclusion, medical image analysis is an interdisciplinary discipline of information science and clinical imaging, and the designed network model should be able to be applied in the clinic to truly achieve intelligent scientific diagnosis in addition to obtaining better performance under experimental conditions; however, in the shortcomings such as too little training data and weak anti-interference ability of the model for medical artificial intelligence models, there are still many roads to go in the future [32]. However, with the development of technology, medical artificial intelligence will certainly serve doctors and patients.

## 7. Conclusion

In this paper, a new therapeutic aid system is designed by combining an artificial intelligence attention mechanism algorithm with incremental music teaching, drawing on the connection principle of biological brain neurons and using the mechanism of music to promote brain neural activity. The artificial method can use a large number of samples to explore the deeper features in the images that are not visible to the naked eye to identify the disease and build a model to improve the accuracy of diagnosis and effectively reduce the phenomenon of misdiagnosis and omission, while the incremental music teaching can soothe the patient's emotion, promote the patient's brain activity, and effectively relieve the patient's condition. In this paper, we designed two network models, Attention Context U-Net and Multidimensional Cross-Attention U-Net, for the automatic segmentation of MS lesions, and the segmentation performance obtained is better than other MS segmentation models and built a supplementary treatment system for MS lesions. A series of experiments were conducted to verify the accuracy. Compared with the traditional transfer learning method-assisted treatment system, the medical assistance system based on the artificial attention mechanism classification method combined with incremental music teaching not only has high classification and diagnosis accuracy but also has improved time efficiency. In conclusion, these high-precision diagnosis and classification results undoubtedly provide some reference value for further diagnosis and follow-up of MS cases.

The article "Design of an Incremental Music Teaching and Assisted Therapy System Based on Artificial Intelligence Attention Mechanism" was retracted in 2023. Reasons: signs of a paper mill; suspected computer-generated content; unreliable results or conclusions; lack of ethics approval or compliance.

## Figures and Tables

**Figure 1:** Column line diagram clinical decision curve.

**Figure 2:** Schematic diagram of the Pearson correlation coefficient.

**Figure 3:** AUC values of the mildly mixed model compared with the mixed model.

**Table 1:** Multifactor logistic regression analysis of the two groups of patients in the training set.

Variable		Reference
Gender	Male	108
	Female	136
Age		25~35
Irregular	No	90
	Yes	154
MS height	Low	14~21
	Middle	21~28
	High	28~35
MS tumor neck width	Low	0.13~0.22
	Middle	0.22~0.31
	High	0.31~0.4
MS irregularity		73
A1 dominance sign		15

**Table 2:** Clinical information of patients in the training set, internal test set, and external test set.

Variable	Training set	Internal test sets	External test sets
Age	25~35	25~35	25~35
EOC percentage	1 : 1.034	1 : 1.134	1 : 1.119
Relapsing remitting	213	201	193
Secondary-progressive	43	51	57
Primary-progressive	26	34	37
Progressive-relapsing	23	19	18

**Table 3:** Features used by different models and their weights.

Features	DWI	ADC	CE-T1W
Mononuclear cell	40	40.866	0.866
Oligoclonal bands	80	81.256	1.256
VEP	120	119.342	-0.658
BAEP	160	161.864	1.864
SEP	200	199.066	-0.934
CSF	240	239.874	-0.126
RGC	280	281.798	1.798
ARV	320	320.826	0.826
MKI	360	361.356	1.356
APV	400	399.574	-0.426

The article "Design of an Incremental Music Teaching and Assisted Therapy System Based on Artificial Intelligence Attention Mechanism" was retracted in 2023. Reasons: signs of a paper mill; suspected computer-generated content; unreliable results or conclusions; lack of ethics approval or compliance.

## Data Availability

The data used to support the findings of this study are available from the corresponding author upon request.
